The article "Secretome of endothelial progenitor cells from stroke patients promotes endothelial barrier tightness and protects against hypoxia-induced vascular leakage" was retracted in 2024. Reason: errors in the cell lines or tissues.

# Secretome of endothelial progenitor cells from stroke patients promotes endothelial barrier tightness and protects against hypoxia-induced vascular leakage

**DOI:** 10.1186/s13287-021-02608-y

**Published:** 2021-10-26

**Authors:** Rodrigo Azevedo Loiola, Miguel García-Gabilondo, Alba Grayston, Paulina Bugno, Agnieszka Kowalska, Sophie Duban-Deweer, Eleonora Rizzi, Johan Hachani, Yasuteru Sano, Fumitaka Shimizu, Takashi Kanda, Caroline Mysiorek, Maciej Piotr Mazurek, Anna Rosell, Fabien Gosselet

**Affiliations:** 1 UR 2465, Blood-Brain Barrier Laboratory (LBHE), Univ. Artois, 62300 Lens, France; 2 Neurovascular Research Laboratory, Vall d’Hebron Institut de Recerca, Universitat Autònoma de Barcelona, 08035 Barcelona, Catalonia Spain; 3 Pure Biologics S.A., Duńska 11, 54-427 Wroclaw, Poland; 4 Department of Neurology and Clinical Neuroscience, Graduate School of Medicine, Yamaguchi University, Ube, Japan; 5 Laboratory of the Blood-Brain Barrier, Sciences Faculty Jean Perrin, Artois University, Lens, France

**Keywords:** Endothelial progenitor cells, Secretome, Blood–brain barrier, Stroke, Angiogenesis, Cell therapy, Cardiovascular disease, Regenerative medicine

## Abstract

**Background:**

Cell-based therapeutic strategies have been proposed as an alternative for brain repair after stroke, but their clinical application has been hampered by potential adverse effects in the long term. The present study was designed to test the effect of the secretome of endothelial progenitor cells (EPCs) from stroke patients (scCM) on in vitro human models of angiogenesis and vascular barrier.

**Methods:**

Two different scCM batches were analysed by mass spectrometry and a proteome profiler. Human primary CD34^+^-derived endothelial cells (CD34^+^-ECs) were used for designing angiogenesis studies (proliferation, migration, and tubulogenesis) or in vitro models of EC monolayer (confluent monolayer ECs—CMECs) and blood–brain barrier (BBB; brain-like ECs—BLECs). Cells were treated with scCM (5 μg/mL) or protein-free endothelial basal medium (scEBM—control). CMECs or BLECs were exposed (6 h) to oxygen–glucose deprivation (OGD) conditions (1% oxygen and glucose-free medium) or normoxia (control—5% oxygen, 1 g/L of glucose) and treated with scCM or scEBM during reoxygenation (24 h).

**Results:**

The analysis of different scCM batches showed a good reproducibility in terms of protein yield and composition. scCM increased CD34^+^-EC proliferation, tubulogenesis, and migration compared to the control (scEBM). The proteomic analysis of scCM revealed the presence of growth factors and molecules modulating cell metabolism and inflammatory pathways. Further, scCM decreased the permeability of CMECs and upregulated the expression of the junctional proteins such as occludin, VE-cadherin, and ZO-1. Such effects were possibly mediated through the activation of the interferon pathway and a moderate downregulation of Wnt signalling. Furthermore, OGD increased the permeability of both CMECs and BLECs, while scCM prevented the OGD-induced vascular leakage in both models. These effects were possibly mediated through the upregulation of junctional proteins and the regulation of MAPK/VEGFR2 activity.

The article "Secretome of endothelial progenitor cells from stroke patients promotes endothelial barrier tightness and protects against hypoxia-induced vascular leakage" was retracted in 2024. Reason: errors in the cell lines or tissues.

**Conclusion:**

Our results suggest that scCM promotes angiogenesis and the maturation of newly formed vessels while restoring the BBB function in ischemic conditions. In conclusion, our results highlight the possibility of using EPC-secretome as a therapeutic alternative to promote brain angiogenesis and protect from ischemia-induced vascular leakage.

**Supplementary Information:**

The online version contains supplementary material available at 10.1186/s13287-021-02608-y.

## Background

Ischemic stroke is among the leading causes of mortality and disability worldwide [1]. In the past decades, recanalization therapy has dramatically reduced the mortality and functional disabilities [1]. However, there are no successful therapies targeting brain repair or vascular remodelling after stroke. Cerebral ischemia results in irreversible damage not only at the neuronal level but also in the brain microvasculature, namely the blood–brain barrier (BBB) [2]. Endothelial cells (ECs) forming a monolayer in brain microvessels are a major component of the BBB, which acts as a physical barrier due to the presence of tight junctions (TJs) between adjacent ECs and the absence of fenestration and pinocytic activity of these cells [3, 4]. Besides, the delivery of essential nutrients to the brain parenchyma is strictly regulated by specific enzymes, receptors, and efflux pumps expressed at the luminal face of the BBB ECs [4]. BBB impairment and vascular disruption are early events following an ischemic stroke, exacerbating the brain injury and contributing to cognitive impairment [2, 5]. In this context, developing new therapies that combine the protection of the BBB integrity and the promotion of angiogenesis could be a potential strategy to improve the functional outcome after stroke. This hypothesis is supported by a body of evidence, suggesting that therapies promoting angiogenesis can stimulate neurogenesis and improve brain repair after stroke [6].

Over the last years, cell therapy with endothelial progenitor cells (EPCs) has been proposed as an alternative approach to promote angiogenesis and brain repair after stroke. EPCs constitute a pool of circulating bone marrow-derived cells that are mobilized towards the damaged tissues after an ischemic injury, where they promote angiogenesis through their incorporation into the vascular wall and the secretion of growth factors [7]. Although several pre-clinical studies have demonstrated that EPCs potentiate neurogenesis and angiogenesis in mouse models of stroke [8–10], the clinical translation of cell-based therapies still raises safety concerns due to their potential adverse side effects [11]. For this reason, clinical trials investigating the potential benefits of cell therapies for ischemic stroke are scarce [12]. In particular, one randomized phase I/IIa clinical trial (NCT01468064) testing the intravenous injection of autologous EPCs for acute stroke [13] did not show serious adverse effects or allergic reactions related to the treatment. In this context, previous studies have reported that the administration of EPC-conditioned medium (EPC-secretome) promotes a beneficial response in pre-clinical models of cerebral ischemia and hypoperfusion [14, 15]. Despite these promising results, mainly obtained with animal cells and models, very few studies have been designed to characterize the effects of EPC-secretome on human cells, in particular in angiogenesis and barrier properties of ECs. The present study was therefore designed to evaluate the effect of EPC-secretome from stroke patients on in vitro models of angiogenesis and ischemia using primary human ECs. Our findings suggest that EPCs from stroke patients produce modulatory molecules which promote angiogenesis and vessel maturation while preventing the hypoxia-induced vascular leakage in oxygen–glucose deprivation (OGD) conditions in vitro. Altogether these data support the use of EPC-secretome to improve microvascular repair in the human brain after stroke.

The article "Secretome of endothelial progenitor cells from stroke patients promotes endothelial barrier tightness and protects against hypoxia-induced vascular leakage" was retracted in 2024. Reason: errors in the cell lines or tissues.

## Methods

### Reagents

EC medium (ECM) and EC growth supplement (ECGS) were purchased from Sciencell (USA); foetal bovine serum (FBS) from Gibco (France); Dulbecco’s modified Eagle medium (DMEM), vascular endothelial growth factor receptor 2 (VEGFR2) kinase inhibitor VII, AKT inhibitor VIII, UO126 monoethanolate, AZ6102, and fibroblast growth factor (FGF) receptor tyrosine kinase inhibitor were purchased from Sigma-Aldrich (France).

### EPC-secretome production

#### EPC-isolation and culture

The EPCs’ isolation from stroke patients and healthy donors was performed as previously described [16]. Frozen EPCs were previously obtained from peripheral blood of both stroke patients (SP: 1—man, 66 years; 2—man, 77 years; 3—woman, 61 years) and healthy donors (HD: 1-woman, 43 years; woman, 39 years; man, 59 years). All donors (stroke or healthy) did not present any known malignant, infectious, or neurological disease (other than the stroke), which were exclusion criteria for the EPC collection. Briefly, blood was collected in EDTA tubes by venous puncture, and Ficoll gradient (1.078 g/L) was used to isolate human mononuclear cells. Isolated cells were seeded on human fibronectin (hFN)-coated 12-well plates at a density of 10^7^ cells/well, cultured with EGM-2 in a 5% CO_2_ incubator at 37 °C. After 3 days in culture, non-adherent cells were discarded and the medium was changed every other day. Colonies of outgrowth ECs appeared between 10 and 20 days after seeding and were further expanded. Immunophenotyping of EPCs was confirmed by von Willebrand factor (vWF—Dako), Ulex Europaeus Agglutinin—1 (UEA-1—Sigma-Aldrich), CD34 (Santa Cruz) and VEGFR2 (Santa Cruz). For EPCs seeding, all flasks were previously pre-coated (37 °C, 45 min) with hFN (1:100) diluted in H_2_O.

#### Low-scale production (LSP) of EPC-secretome

The LSP was performed to obtain small quantities of EPC-secretome from both stroke patients and healthy donors as usually performed in academic laboratories for studying EPCs. Briefly, EPCs (3 × 10^6^ cells) from HD and SP were resuspended in 12 mL of complete EGM-2 and seeded in T75 flasks (75 cm^2^). After 72 h, cells were rinsed (PBS-CMF) and incubated (1 h) with DMEM. Then, DMEM was discarded and cells were cultivated with 12 mL of endothelial basal medium (EBM—Lonza) without the addition of any supplements. After 24 h, the conditioned medium (HD-CM or SP-CM) was collected.

#### High-scale production (HSP) of EPC-secretome

The HSP was performed in 10-layer culture flasks to provide higher content of proteins in the conditioned medium, which is desirable to consider future studies and treatments in patients. Briefly, EPCs (1 × 10^7^ cells) from SP-1 donor were resuspended in 25 mL of EGM-2 and seeded in a T175 flask (175 cm^2^). After 96 h, EPCs were trypsinized and split in three T300 flasks (300 cm^2^). For every T300 flask, 2 × 10^7^ cells were seeded in 70 mL of complete EGM-2 medium. After 72 h, EPCs were trypsinized, resuspended (2.48 × 10^8^ cells) in 1 L of EGM-2, and seeded in a CF10 flask (Nunc™ EasyFill™ Cell Factory™ Systems, culture area 6320 cm^2^). After 96 h (100% confluence), the EGM-2 medium was discarded and cells were rinsed with PBS-CMF. Next, cells were incubated in DMEM medium, which was discarded after 1 h and replaced with 1L of EBM without supplements. After 24 h, CM was collected and filtered/concentrated.

#### Filtration and concentration of EPC-secretome

EPC-secretome obtained by LSP (HD-CM and SP-CM) or HSP (CM), and fresh protein-free EBM (control) were filtered through a 0.22-μm vacuum filter to remove cells and debris. Centricon Plus-70 filters (3 kDa Ultracel-PL membrane—Millipore) were filled with EPC-secretome or EBM and centrifuged (3500×g) at 4 °C for 60 min. The super-concentrated EPC-secretomes (scHD-CM, scSP-CM, scCM) or EBM (scEBM) was recovered by centrifuging in collection mode at 1000 g for 1 min. Finally, the protein content was determined by Bradford assay and frozen at − 80 °C in low-protein binding tubes.

The article "Secretome of endothelial progenitor cells from stroke patients promotes endothelial barrier tightness and protects against hypoxia-induced vascular leakage" was retracted in 2024. Reason: errors in the cell lines or tissues.

### Treatments

All experiments were performed in the absence of serum or other commercial growth factors. The EPC-secretome (5 μg/mL of either scSP-CM, scHD-CM, or scCM) or scEBM (control) was diluted in serum-free ECM containing bovine serum albumin (BSA) 0.1%. For the experiments using inhibitors, CD34^+^-ECs were pre-treated 30 min before adding scEBM or scCM using the following concentrations: UO126 (MAPK inhibitor—1 μmol/L); VEGFR2 kinase inhibitor VII (10 μmol/L); AKT inhibitor VIII (1 μmol/L); AZ6102 (Wnt inhibitor-1 μmol/L); FGFR tyrosine kinase inhibitor (1 μmol/L). For experiments using TNFα cells were pre-treated (24 h) with scCM or scEBM, and then, TNFα (10 ng/mL—Sigma-Aldrich) was added. After 24 h, a permeability assay and sample collection were performed.

### Cells

CD34^+^ cells were isolated from human umbilical cord blood and differentiated into ECs (CD34^+^-ECs), as previously described [17]. CD34^+^-ECs were seeded in 100-mm 1% gelatin-coated dishes with ECM-containing ECGS and 5% FBS (named ECM5). After two days, cells were trypsinized and seeded for the experiments of angiogenesis (cell proliferation, tubulogenesis, and migration) or the preparation of CMECs and BLECs, as further described.

For the co-culture approach (in vitro BBB model), human–brain pericytes (HBPs) were grown in DMEM containing 4.5 g/L D-glucose, 10% FBS, 1% L-glutamine, and 1% penicillin–streptomycin, as previously described [18, 19].

### Cell proliferation

CD34^+^-ECs were seeded (5 × 10^3^ cells/well) in 1% gelatin-coated 96-well plates. After 24 h, CD34^+^-ECs were serum-starved in ECM with 0.1% BSA for 6 h. Then, cells were treated (24 h) with EPC-secretome (scHD-CM, scSP-CM, or scCM) or scEBM. Cell viability was evaluated by a resazurin assay, as previously reported [20]. ATP levels were measured with a luminescent kit (CellTiter Glo™, Promega, France) following the manufacturer’s instructions (Additional File 1: Figure S1). To assess the effect of the treatment on cell proliferation/growth, CD34^+^-ECs were seeded at a low density, and the experiments were performed during the exponential growth phase, when no cell death was observed. Cell proliferation thus represents the cell viability (relative number of living cells) of EPC-secretome-treated CD34^+^-ECs compared to scEBM-treated cells. Cell proliferation data were represented as the relative percentage versus the scEBM (control) group.

The article "Secretome of endothelial progenitor cells from stroke patients promotes endothelial barrier tightness and protects against hypoxia-induced vascular leakage" was retracted in 2024. Reason: errors in the cell lines or tissues.

### Wound healing assay

CD34^+^-ECs (2 × 10^5^ cells/well) were seeded in 1% gelatin-coated 24-well plates. After 24 h, CD34^+^-ECs were serum-starved in ECM with 0.1% BSA for 6 h. Then, a wound was created by scratching the cell monolayer with a 200-μL tip. Cells were rinsed with DMEM to remove cell debris and treated with EPC-secretome (scHD-CM, scSP-CM, or scCM) or scEBM. Images of the wound were taken immediately after the scratch (time 0) and 16 h after the treatments using a phase-contrast microscope (Nikon). The wound healing of EPC-secretome-treated cells was calculated by measuring the difference between the initial (time 0) and final (time 16 h) wound area using the ImageJ software. The migration of EPC-secretome-treated CD34^+^-ECs was calculated as the relative percentage compared to the scEBM-treated cells.

### Capillary-like tubulogenesis assay

Angiogenesis μ-slides (IBIDI, Germany) were coated with Matrigel™ (BD Biosciences—10 μL/well) and incubated at 37 °C for 1 h, as previously described [21]. After serum-starvation (ECM + 0.1% BSA) for 16 h, CD34^+^-ECs were detached and seeded (12 × 10^3^ cells/well) on the surface of polymerized Matrigel™ and treated with EPC-secretome (scSP-CM, scHD-CM, scCM) or scEBM. After 6-h incubation, pictures were taken using a phase-contrast microscope (Nikon) with a 5 × magnification objective. The number of tubular structures was determined using the Wimasis® Image Analysis software , and the tubulogenesis of EPC-secretome-treated CD34^+^-ECs was calculated as the relative percentage versus the scEBM-treated cells.

### Confluent monolayers of endothelial cells (CMECs)

Briefly, CD34^+^-ECs (8 × 10^4^ cells/insert) were seeded in Matrigel™-coated Transwell inserts (Costar Transwell inserts, pore size 0.4 μm). Filters were placed in 12-well plates containing ECM5, and after 4 days, cells were treated with scCM or scEBM. Then, 48 h later, permeability studies and sample collection were performed.

### In vitro BBB model with brain-like endothelial cells (BLECs)

The BBB model was reproduced as previously published [22]. Briefly, CD34^+^-ECs (8 × 10^4^ cells/insert) were seeded into Matrigel™-coated filters (Costar Transwell inserts, pore size 0.4 μm). Then, inserts were placed in collagen-coated 12-well plates containing HBPs (5 × 10^4^ cells/well). After 5 days of co-culture, CD34^+^-ECs acquire the major BBB properties observed in vivo [23] and reproduce a suitable model to investigate BBB permeability and physiology [22, 24]. They are therefore named as brain-like ECs (BLECs). Once differentiated, BLECs were treated with scCM or scEBM and, 48 h later, permeability studies and sample collection were performed.

The article "Secretome of endothelial progenitor cells from stroke patients promotes endothelial barrier tightness and protects against hypoxia-induced vascular leakage" was retracted in 2024. Reason: errors in the cell lines or tissues.

### Permeability assay

Permeability assays were performed as previously described [25]. HEPES-buffered Ringer’s solution was added to empty wells in a 12-well plate (Costar). Filter inserts containing CMECs or BLECs were subsequently placed in the 12-well plate and filled with Ringer-Hepes buffer (RH) containing the fluorescent integrity marker sodium fluorescein (Naf; 10 µM; Life Technologies), which poorly crosses the BBB. Alternatively, some experiments were performed with radiolabeled sucrose-C^14^, another paracellular marker that also poorly crosses the BBB (Additional file 2: Figure S2a). After 1 h, filter inserts were withdrawn from the receiver compartment. Aliquots from the donor solution were taken at the beginning and the end of the experiments, and the fluorescence was quantified. The permeability coefficient was calculated as previously described [26]. Briefly, both insert permeability (PSf, for insert only coated with Matrigel™) and permeability of inserts containing either CMECs or BLECs (PSt, for insert with Matrigel™ and cells) were considered, according to the following formula: 1/PSe = 1/PSt − 1/PSf. The permeability value for the CMECs’ or BLECs’ monolayer was then divided by the surface area of the insert (1.12 cm^2^) to obtain the permeability coefficient (Pe) of each molecule (cm/min).

### Immunofluorescence

Cells were fixed with cold methanol and rinsed twice with cold PBS-CMF. Unspecific binding was blocked (30 min, RT) using a Sea Block buffer solution (Thermo Fisher Scientific). Then, cells were incubated (60 min, RT) with the primary antibodies against claudin 5 (Invitrogen, 34-1600), ZO-1 (Invitrogen, 61-7300), VE-cadherin (Abcam, Ab33168), or occludin (Invitrogen, 71-500) in PBS-CMF containing 2% (v/v) normal goat serum (PBS-NGS). After rinsing, cells were incubated (30 min, RT) with a secondary polyclonal antibody (Life Technologies, A-11034). For F actin staining, cells were fixed with 4% paraformaldehyde (PFA) and permeabilized using Triton 0.1% in PBS-CMF (10 min, RT). Then, cells were incubated (30 min, RT) with phalloidin (Bodipy—588/568—Thermo Fisher, B3475) diluted in PBS-NGS. After rising, cells were mounted using ProLong Gold antifade mountant (Thermo Fisher) containing DAPI (nuclear staining). Images were acquired using a Leica microscope (DMRD; Leica Microsystems) and processed using the ImageJ software.

### qPCR

The mRNA from cells was extracted using the NucleoSpin® RNA/protein kit (Macherey–Nagel, Germany). cDNA was obtained from 250 ng of mRNA using IScript™ Reverse Transcription Supermix (BioRad, USA), following the manufacturer’s instructions. qPCRs (10 µL) were prepared using SsoFast™ EvaGreen® Supermix (BioRad), primers (100 nM), deionized water, and cDNA. qPCR amplification was carried out for 40 cycles with an annealing temperature of 60 °C in a CFX96 thermocycler (BioRad). Ct data were obtained using the Bio-Rad CFX Manager software. Gene expression levels of the targets (Table 1) were calculated using the 2^-^^ΔΔCt^ method, relative to the housekeeping gene *PPIA* (Cyclophilin A).

The article "Secretome of endothelial progenitor cells from stroke patients promotes endothelial barrier tightness and protects against hypoxia-induced vascular leakage" was retracted in 2024. Reason: errors in the cell lines or tissues.

**Table 1:** List of primers used in the study and their corresponding sequence

Target	Gene	Primer sequence
Cyclin D1	***CCND1***	Forward: GAAGATCGTCGCCACCTGGA
		Reverse: CAGGCGGCTCTTTTTCACGG
APC Downregulated 1	***APCDD1***	Forward: ACTGATGCCACCCAGAGGATG
		Reverse: AGATGATCCGACAGGCGATGC
Axin 2	***Axin 2***	Forward: CCTGGGGGCAGCGAGTATTA
		Reverse: TTGGGCAAGGTACTGCCTCT
Vascular endothelial growth factor A	***VEGFA***	Forward: AGAAGGAGGAGGGCAGAATC
		Reverse: ACACAGGATGGCTTGAAGATG
Cyclophilin A	***PPIA***	Forward: CTGAGGACTGGAGAGAAAGGAT
		Reverse: GAAGTCACCACCCTGACACATA
Glucose transporter 1 (GLUT1)	***SLC2A1***	Forward: CTTCTCCAACTGGACCTCAAAT
		Reverse: AGGAGCACAGTGAAGATGATGA
Hypoxia-induced factor 1α (HIF1α)	***HIF1A***	Forward: GGATCAGACACCTAGTCCTT
		Reverse: ATCCATTGGGATATAGGGAG

### Western blotting (WB)

Cells were collected with RIPA lysis buffer containing protease and phosphatase inhibitors (Sigma-Aldrich). Cell lysates (10–20 μg) were prepared, placed on sodium dodecyl sulphate–polyacrylamide gel electrophoresis (SDS-PAGE) and then transferred to nitrocellulose membranes (GE Healthcare, Germany). Non-specific binding was blocked using tris-buffered saline containing 0.1% Tween 20 (TBS-T) with 5% of skimmed milk (1 h, RT). Membranes were incubated (4 °C, overnight) with primary antibodies (Table 2), washed extensively and then incubated (1 h, RT) with a horseradish peroxidase-conjugated secondary antibody (Dako/Agilent Technologies). After rinsing, membranes were developed with a chemiluminescence reagent (GE Healthcare), and images were acquired using the WB Imaging System Azure c600 (Azure BioSystems). The software TotalLab TL 100 1D gel Analysis was used for quantification of the relative immunoblots densities. Conditions and concentrations of each antibody shown in Table 2 were previously optimized, as demonstrated in Additional file 3: Figure S3. Western blot images shown in this study were cropped, but original results obtained for each experiment performed are provided in Additional file 4: Figure S4, Additional file 5: Figure S5, Additional file 6: Figure S6, Additional file 7: Figure S7, Additional file 8: Figure S8, Additional file 9: Figure S9, Additional file 10: Figure S10, Additional file 11: Figure S11, Additional file 12: Figure S12, Additional file 13: Figure S13. More pictures and data can be provided upon request.

The article "Secretome of endothelial progenitor cells from stroke patients promotes endothelial barrier tightness and protects against hypoxia-induced vascular leakage" was retracted in 2024. Reason: errors in the cell lines or tissues.

**Table 2:** List of antibodies used in the study

Target	Reference	Provider
COX-2	AF4198	R&D Systems
Phospho-VEGFR2	AF1766	R&D Systems
Phospho-AKT	MAB887	R&D Systems
pan-VEGFR2	sc6251	SantaCruz
Non-phospho(active)-β catenin	19,807	CellSignalling
Phospho-ERK1/2	9106	CellSignalling
pan-ERK1/2	9102	CellSignalling
pan-AKT	4691	CellSignalling
pan-β catenin	Ab6302	Abcam
BCRP	Ab3380	Abcam
ICAM-1	Ab53013	Abcam
VCAM-1	Ab98954	Abcam
Tricellulin	Ab253067	Abcam
ABCA1	Ab18180	Abcam
β-actin	A5541	Sigma Aldrich
P-gp	C219	Genetex
VE-cadherin	Ab33168	Abcam
ZO-1	Ab216880	Abcam
Claudin 5	Ab15106	Abcam
Occludin	Ab31721	Abcam

### In vitro oxygen–glucose deprivation (OGD) assay

The in vitro OGD model was designed to simulate the in vivo stroke conditions, with a shortage of oxygen (1% O_2_) and nutrients (glucose-free medium), which were achieved by using a hypoxic chamber (Whitley H35 Hypoxistation). In parallel, experiments performed under normoxic conditions (5% CO_2_/95% air and 1 g/L glucose) were used as controls. All media and solutions used for the OGD conditions were previously equilibrated in the hypoxic chamber. Then, inserts were submitted to OGD or normoxic conditions for 6 h and permeability assays or sample collection were performed. In another set of inserts, cells exposed to OGD or normoxic conditions were treated with scCM or scEBM and submitted to a reoxygenation phase (24 h), which consists in returning the cells to physiological conditions, thereby mimicking the in vivo reperfusion phase. After reoxygenation, permeability assay and sample collection were performed.

### scCM protein profile

The protein content was analysed in two independent batches of scCM using the Proteome Profiler Human Angiogenesis Array kit (R&D Systems, USA), which can detect the expression of 55 angiogenesis-related proteins. Briefly, scCM (150 μg of total protein) was mixed with the biotinylated detection antibodies provided in the kit and incubated (4 °C, overnight) in a nitrocellulose membrane containing the capture antibodies. After incubation, the membranes were washed and the Streptavidin-HRP and chemiluminescent detection reagents were applied. The spot signal was detected with the Luminescent Imaging System Azure c600 (Azure Biosystem), and quantification of the relative densities of the bands was performed using the TotalLab TL 100 1D gel Analysis software. scEBM was used as a negative control. Results are expressed as the percentage of the signal relative to the reference spot (loading control).

The article "Secretome of endothelial progenitor cells from stroke patients promotes endothelial barrier tightness and protects against hypoxia-induced vascular leakage" was retracted in 2024. Reason: errors in the cell lines or tissues.

### Proteomic analysis of scCM

#### Preparation of the samples

Proteins were extracted from two independent batches of scCM (~ 100 µg each) in a 1.5 M Tris–HCl buffer (pH 8.5) containing 7 M guanidine hydrochloride (GuHCl), 20 mM ethylenediaminetetraacetate (EDTA), and 0.5 M dithiothreitol (DTT), and incubated for 1 h at 60 °C. The sulfhydryl groups of the proteins were carbamidomethylated with iodoacetamide used in a 2.5-fold excess (w/w) to DTT in the dark (20 min, RT). The suspension was centrifuged at 11.000 g for 15 min at 4 °C, and the supernatant was collected. Protein concentration was measured using the Quick start Bradford dye reagent (Biorad, Hercules, USA) with BSA as a standard protein. For each sample, 100 μg of protein was precipitated in 80% acetone overnight at − 20 °C. After 15 min of centrifugation at 11.000 g, the pellet was enzymatically digested overnight using a sequencing grade modified trypsin (Promega, Madison, USA) with an enzyme/substrate ratio of 1/50 at 37 °C in 25 mM ammonium bicarbonate (NH_4_HCO_3_). The reaction was stopped by adding formic acid to a final concentration of 0.1% (v/v). Peptides were extracted using the HyperSep SpinTip Microscale C18 (Thermo Fisher Scientific, USA), and the peptides’ concentration was measured using the Quantitative Colorimetric Peptide Assay (Thermo Fisher Scientific, USA).

### Data-dependent acquisition by mass spectrometry (DDA-MS)

DDA consists in a proteomic approach in which digested peptides are ionized and analysed by MS. Peptide signals that raised in a full-scan mass spectrum with predefined MS parameters were selected for fragmentation, and then, their tandem product (MS/MS) mass spectra were matched to spectra in a protein database. Briefly, two micrograms of peptides from each sample was analysed using an Eksigent nano-LC 2D HPLC system connected to a quadrupole time-of-flight Triple TOF 5600 + mass spectrometer (Sciex, Redwood City, USA). After injection, peptide mixtures were transferred into a nano-HPLC column (ChromXP C18, 3 μm 120 A, nanoLC column, 3C18-CL, 75 μmx15cm, Sciex, USA) at a flow rate of 300 nL/min using the following gradients for solvent B: 2 to 8% solvent B in A (from 0 to 5 min), 8 to 35% B (5 to 90 min), 35 to 40% B (90 to 100 min), 40 to 90% B (100 to 102 min), 90% B (102 to 107 min), 90 to 2% B (107 to 109 min) and finally 2% solvent B in A (109 to 140 min), with a total runtime of 140 min including a mobile phase equilibration. The following solvents were added in the mobile phase A: 2% acetonitrile/98% of 0.1% formic acid (v/v) in water; and in the mobile phase B: 98% acetonitrile/2% of 0.1% formic acid (v/v) in water. The eluted peptides were directly injected for MS data acquisition in a hybrid quadrupole-TOF 5600 + System fitted with a Nanospray III source. Ionization was obtained with an ion spray voltage of 2.2 kV, curtain gas set at 25 psi, and ion source gas at 3 psi, using positive-ion mode. DDA-MS survey scans were acquired at 250 ms from 400 to 1500 *m*/*z* and MS/MS scan from 100 to 2000 *m*/*z* (100 ms accumulation time, 50 mDa mass tolerance, rolling collision energy).

The article "Secretome of endothelial progenitor cells from stroke patients promotes endothelial barrier tightness and protects against hypoxia-induced vascular leakage" was retracted in 2024. Reason: errors in the cell lines or tissues.

Peptide and protein identifications were performed using the Protein Pilot software (version 5.0.2, Sciex) with a Swiss-Prot/TrEMBL concatenated target-reverse decoy database (downloaded in November 2018), specifying iodoacetamide and methionine oxidation as variable modifications. The false discovery rate (FDR) was used to generate a spectral library and was set to 1% for both peptides and proteins.

### TempO-Seq analysis

Targeted transcriptome quantification assay (TempO-Seq, BioSpyder) was performed in CMECs (*n* = 3 per group) treated with scCM (5 μg/mL) or scEBM (control). Cells were rinsed with sterile PBS-CMF, lysed using a TempO-Seq lysis buffer, and stored at − 80° C before shipment to BioClavis (Glasgow, UK), where the TempO-Seq assay was performed. The TempO-Seq analysis was performed as previously described [27]. Briefly, the toxicity pathway analysis was performed using a list of genes annotated to different stress response pathways (3565 probe-set representing 3257 genes). The FASTQ file from each sample was aligned against the TempO-Seq transcriptome using the Bowtie aligner, generating a table of counts per gene and sample, which was further analysed using the R software. The differential expression analysis was performed by comparing the scCM-treated samples with their suitable control (scEBM). Genes were considered significantly differentially expressed when the Benjamin Hochberg adjusted *P* value was < 0.05.

### Statistical analysis

All statistics were analysed using GraphPad Prism® software version 6.0. The normality of continuous variables was assessed using the Shapiro–Wilk test (*n* < 30) or Kolmogorov–Smirnov test (*n*  ≥ 30). For variables that were not normally distributed, Mann–Whitney or Kruskal–Wallis tests were performed and the values were expressed as median (interquartile range 25–75). For variables that were normally distributed, Student’s t test or one-way ANOVA followed by Tukey's multiple comparisons test was performed, and the values were expressed as mean ± standard deviation (SD). The threshold for statistical significance was set as *P* < 0.05 (*).

The article "Secretome of endothelial progenitor cells from stroke patients promotes endothelial barrier tightness and protects against hypoxia-induced vascular leakage" was retracted in 2024. Reason: errors in the cell lines or tissues.

## Results

### EPC-secretome from stroke patients promotes in vitro angiogenesis

Previous studies have reported conflicting findings regarding the effect of cardiovascular diseases in the function of EPCs [10, 28]. Therefore, we initially compared the angiogenic properties of EPC-secretome from three stroke patients (scSP-CM) and three healthy donors (scHD-CM) using LSP conditions in CD34^+^-EC. Our results suggest that scSP-CM preserves their angiogenic properties, as they showed a similar effect on CD34^+^-ECs proliferation (scHD-CM: 131.5% [129.3–139.9] and scSP-CM: 141.4% [133.4–146.5]) (Fig. 1a) and migration (scHD-CM: 461.6% [385.4–534.8] and scSP-CM: 340.3% [310.4–699.1]) (Fig. 1b) compared to scHD-CM, whereas neither scHD-CM nor scSP-CM had any effect on tubulogenesis (Fig. 1c).

**Fig. 1:** EPC-secretome from stroke patients promotes in vitro angiogenesis. EPC-secretome obtained from stroke patients (scSP-CM) and healthy donors (scHD-CM) under low-scale production conditions have similar effects on CD34^+^-ECs proliferation (**a**), migration (**b**), and tubulogenesis (**c**). Further, EPC-secretome obtained from stroke patients produced at high-scale conditions (scCM) increased CD34^+^-ECs proliferation (**d**), migration (**e**), and tubulogenesis (**f**). Besides, two scCM batches were compared and showed similar effects (scCM-1, batch 1; scCM-2, batch 2). The effects of scCM were similar to those observed with VEGF-A (50 ng/mL). Data represent median (interquartile range) (*n* = 3–8), *P < 0.05 vs scEBM. Scale bar: 200 μm

Then, we developed a method to obtain EPC-secretome from stroke patients under HSP conditions (scCM), which provided a higher yield of protein content (168-fold increase) in comparison with LSP conditions (LSP: 207 ± 13.6 μg vs HSP: 34.9 ± 1.6 mg). scCM promoted a consistent increase on CD34^+^-EC proliferation (139.6% [134.8–183.4]) (Fig. 1d), migration (264.3% [203.4–349.6]) (Fig. 1e), and tubulogenesis (120.7% [103.3–142.4]) (Fig. 1f), which was similar to the results observed with VEGF-A. Besides, we observed similar effects when comparing two different scCM batches (scCM-1 and scCM-2). The positive effect of scCM-1 and scCM-2 on CD34^+^-ECs viability was further confirmed by measuring the ATP content, a complementary assay for measuring cell viability (Additional file 1: Fig. 1).

### scCM characterization

A multiplex antibody assay was performed for the detection of angiogenesis-related proteins in two scCM batches. Among the investigated targets [55], we detected the presence of 20 proteins involved in angiogenesis (Fig. 2a), including growth factors such as VEGF-A, FGF, angiogenin, and platelet-derived growth factor (PDGF). Moreover, we detected the presence of molecules involved in inflammatory responses (interleukin 8—IL8; CXCL16; Serpin E1) and modulators of extracellular matrix degradation (metalloproteinase 9—MMP9; tissue inhibitor of metalloproteinase 1 and 4—TIMP1 and TIMP4; urokinase-type plasminogen activator—uPA). Interestingly, we detected consistent levels of Serpin F1 and thrombospondin, which are well known to play an anti-angiogenic activity [29, 30]. Next, a DDA-MS analysis of two scCM batches revealed 1041 common proteins (Fig. 2b). By using the Panther software (Protein Analysis THrough Evolutionary Relationships, version 16.0), such proteins were converted in gene identifiers and were then classified according to their protein class (Fig. 2c), molecular function (Fig. 2d), and biological process (Fig. 2e). Besides, a Gene Ontology (GO) enrichment analysis revealed an overrepresentation (fold enrichment) of pathways involved in cell metabolism, such as serine glycine biosynthesis, pentose phosphate pathway, glycolysis, pyruvate metabolism, and TCA cycle (Fig. 2f and Additional file 14: Table S1).

The article "Secretome of endothelial progenitor cells from stroke patients promotes endothelial barrier tightness and protects against hypoxia-induced vascular leakage" was retracted in 2024. Reason: errors in the cell lines or tissues.

**Fig. 2:** Identification of proteins in scCM. Detection of pro-angiogenesis factors in two batches of scCM was performed by Angiogenesis Proteome Profiler (**a**). Two different batches of scCM were analysed by MS. Over 1200 proteins were identified and the two batches of scCM shared 1041 proteins (**b**). The set of proteins shared between two batches of scCM (1041) were converted in gene identifiers and then submitted to an enrichment analysis using the GeneOntology/Panther software. The proteins were classified according to protein class (**c**), molecular (**d**), or biological function (**e**). Among the Panther pathways that were over-represented in the enrichment analysis of scCM samples, several were related to cell metabolism (**f**)

### scCM-induced angiogenesis is mediated through MAPK kinase and receptor tyrosine kinase (RTK) activation

To further investigate the underlying mechanisms of the observed scCM-induced effects, we evaluated the activation of MAPK, VEGFR2, and PI3K/AKT signalling pathways, key modulators of angiogenesis. scCM induced a strong and consistent ERK1/2 phosphorylation (scCM, 10 min: 2599% [1102–2723]), whereas it did not affect either AKT or VEGFR2 phosphorylation (Fig. 3a). Further, we observed that ERK1/2 activation lasts for at least 4 h, getting normalized after 24 h of treatment (Fig. 3b). Interestingly, AKT activation is reduced at 4 and 24 h after scCM treatment, while VEGFR2 phosphorylation is increased after 24 h of treatment (Fig. 3b). Inhibition of ERK pathway (using UO126), VEGFR2 (using VEGFR kinase inhibitor VII), and FGF receptor (using FGFR tyrosine kinase inhibitor) attenuated the scCM-induced increase on CD34^+^-EC proliferation (Fig. 3c). Additionally, VEGFR2 and FGFR inhibition reduced the scCM-induced migration (Fig. 3d). The efficiency of ERK1/2 and VEGFR2 inhibition was confirmed by WB (Fig. 3e). STRING analysis database (version 11.0, released 2019.01.19) was used to classify the scCM proteins as involved with “angiogenesis” (8 proteins), “VEGF-A pathway” (4 proteins), and “FGF pathway” (15 proteins). Among them, most were adapter proteins (14–3-3 superfamily and CRK), GTPases (RHOC, RAC1, and RAC3), or serine/threonine-protein phosphatases (PPP2R1A, PP2CA, and PPP2CB). By creating an interaction map among these proteins, we observed that MAPK1 (ERK2) was central in the network hub (Fig. 3f).

The article "Secretome of endothelial progenitor cells from stroke patients promotes endothelial barrier tightness and protects against hypoxia-induced vascular leakage" was retracted in 2024. Reason: errors in the cell lines or tissues.

**Fig. 3:** scCM promotes in vitro angiogenesis mediated by MAPK and VEGFR2 activation. scCM induces a rapid and consistent increase in ERK1/2 phosphorylation, whereas it does not affect AKT or VEGFR2 activation (**a**). ERK1/2 activation remains until 4 h after treatment, while VEGFR2 phosphorylation is upregulated after 24 h of treatment (**b**). Pre-incubation with UO126 (MEK/ERK inhibitor—1 μmol/L), VEGFR2 kinase inhibitor VII (10 μmol/L) and FGFR tyrosine kinase inhibitor (1 μmol/L) reduced the scCM-induced proliferation (**c**) while VEGFR2 and FGFR inhibition reduced the scCM-induced migration (**d**). Western blot detection of ERK1/2 and VEGFR2 phosphorylation on cells treated with either vehicle (DMSO), MEK/ERK1/2, or VEGFR2, or FGFR inhibitors (**e**). Proteins classified as involved in angiogenesis [8], VEGF-A [4], and FGF [15] were grouped, then converted in gene identifiers and an interaction network was prepared using Cytoscape software (version 3.8.2, released 2020.10.24). Such pathways share in common the protein MAPK1 (ERK2) (**f**). Data represent median (interquartile range) (*n* = 3–7), *P < 0.05 vs scEBM; $*P* < 0.05 vs scCM vehicle

### scCM promotes vascular tightness

To understand the effect of scCM on vascular permeability, CMECs were used as a model of newly formed vessels, which presents an elevated permeability in comparison with fully matured BBB microvessels. In parallel, BLECs were used as an in vitro BBB model, characterized by the presence of TJ and an extremely low permeability. Indeed, the crossing of sucrose C^14^, a classical paracellular marker for permeability studies, showed a 2.45-fold increase through CMECs when compared to BLECs (Additional file 2: Figure S2a). Similar results were observed using the fluorescent marker Naf, although the difference between CMECs and BLECs was more discrete (+ 50%) (Fig. 4a). However, given the concerns associated with the manipulation and disposal of radioactive tracers, further experiments were performed with Naf. At such conditions, VEGF-A (50 ng/mL) promoted a consistent increase in the permeability of both CMECs (2.7-fold increase) and BLECs (2.3-fold increase) (Additional file 2: Figure S2b). scCM treatment decreased CMECs permeability (scEBM: 1.03 ± 0.08 × 10^–3^ cm/min vs scCM: 0.76 ± 0.06 × 10^–3^ cm/min), while it did not affect BLECs. WB analysis showed that scCM increases the expression of VE-Cadherin (113.5% [107.3–125.8]), ZO-1 (176% [104.6–209.3]), and occludin (121.1% [115.2–143.9]) in CMECs (Fig. 4b), whereas it had no effect on BLECs. IF analysis suggested that scCM favours the localization of TJ at the cell junctions and decreases its accumulation in the cytoplasm of CMECs (Additional file 2: Figure S2c). Besides, we observed that scCM-treated cells presented an accumulation of F-actin fibres at the cell junctions (Additional file 15: Figure S14a-b). Furthermore, scCM upregulated P-glycoprotein (Pg-p) in BLECs, one of the major efflux pumps of the ABC family restricting xenobiotics entrance into the CNS, while it had no effect in Breast Cancer Resistant Protein (BCRP) and ABC subfamily A member 1 (ABCA1) in neither CMECs nor BLECs (Additional file 15: Figure S14c).

The article "Secretome of endothelial progenitor cells from stroke patients promotes endothelial barrier tightness and protects against hypoxia-induced vascular leakage" was retracted in 2024. Reason: errors in the cell lines or tissues.

**Fig. 4:** scCM promotes endothelial barrier tightness. scCM reduced the permeability of CMECs, while it did not affect BLECs (**a**). scCM upregulated the expression of junctional proteins on CMECs (**b**). Heat map representing 23 genes upregulated by scCM on CMECs, most of them associated with the IFN pathway (**c**). scCM reduced the content of active β-catenin and claudin 3 (**d**) and downregulated mRNA expression of Wnt pathway targets APCDD1, Axin2, and CCND1 on CMECs (**e**). Co-incubation with Wnt inhibitor (AZ6102, 1 μmol/L) decreased barrier permeability of cells treated with scEBM (**f**). Data represent median (interquartile range) [**b**, **d**, and **e**] or mean ± SD [**a** and **f**] (*n* = 4–8). *P < 0.05vs scEBM CMECs

### scCM upregulates the expression of genes involved in the interferon pathway

We further investigated the underlying mechanisms of scCM effects in CMECs by performing an mRNA sequencing by TempO-seq. scCM upregulated the expression of 23 genes (Fig. 4c). By analysing the upregulated genes using the Panther software, we observed an overrepresentation of genes involved in interferon (IFN) pathways (Table 3 and Additional file 16: Table S2) according to the Reactome database. Given that previous studies have suggested that IFN response can inhibit the Wnt pathway activation [31], we investigated the effect of scCM on Wnt signalling. The levels of non-phosphorylated β-catenin, which translocates into the nucleus and transduces the Wnt pathway signalling, were reduced in scCM-treated cells (91.5% [80.8–92.6]) (Fig. 4d) together with a downregulation of claudin 3 (53.7% [48.1–66.2]), a target which is positively correlated with Wnt activation (Fig. 4d). Further, we observed a reduction in the mRNA expression of Wnt pathway targets (APCDD1, Axin 2, CCND1) (Fig. 4e). Besides, Wnt pathway inhibitor (AZ6102, 1 μmol/L) did not affect scCM-treated cells, while it caused a consistent decrease (scEBM vehicle: 100 ± 3.7% vs scEBM AZ6102: 73.2 ± 11.8%) in the permeability of scEBM-treated cells (Fig. 4f).

The article "Secretome of endothelial progenitor cells from stroke patients promotes endothelial barrier tightness and protects against hypoxia-induced vascular leakage" was retracted in 2024. Reason: errors in the cell lines or tissues.

**Table 3:** Pathways overrepresented in CMECs treated with scCM

Reactome Pathways	Homo sapiens (*n*)	scCM (*n*)	scCM (expected)	Fold enrichment	*P*-value
*Interferon alpha/beta signalling (R-HSA-909733)*	67	9	.07	> 100	1.25E−13
*Interferon Signalling (R-HSA-913531)*‬‬‬‬‬‬‬‬‬‬‬‬‬‬‬‬‬‬‬‬‬‬‬‬‬‬	196	9	.22	41.12	1.19E−09
*Cytokine Signalling in Immune system (R-HSA-1280215)*	823	12	.92	13.06	3.34E−08
*Interleukin-10 signalling (R-HSA-6783783)*	45	3	.05	59.70	4.20E−02
*Antiviral mechanism by IFN-stimulated genes (R-HSA-1169410)*	79	4	.09	45.34	4.22E−03

Upregulated genes (23 genes) in scCM-treated CMECs were analysed by the Panther software based on the human database. Pathways (Reactome database) which were overrepresented (fold enrichment) were mainly related to IFN and inflammatory pathways. *N*: number of genes found in the human genome (Homo sapiens) or scCM; Expected: number of genes expected for a certain pathway based on the Reactome database; Fold enrichment: scCM (*n*)/scCM (expected)

### scCM protects against OGD-induced barrier disruption

Next, CMECs and BLECs were exposed to OGD mimicking the conditions observed after stroke. OGD did not affect CMECs (Additional file 17: Figure S15a), while it induced a marked increase in the permeability of BLECs (normoxia: 0.66 [0.63–0.69] vs OGD: 1.18 [0.92–1.25] × 10^–3^ cm/min) (Additional file 17: Figure S15b). Besides, OGD upregulated the expression of hypoxia-target genes (HIF1A, VEGF-A, and GLUT1) in both CMECs and BLECs (Additional file 17: Figure S15c). While we could not detect any marked effect of OGD on TJ expression (Additional file 17: Figure S15d), IF suggested that OGD changed the distribution of junctional proteins (Additional file 17: Figure S15e–f).

To evaluate the protective effect of scCM under ischemic conditions, cells were treated after OGD or normoxia with scEBM or scCM during re-oxygenation (R-normoxia or R-OGD). CMECs exposed to OGD conditions presented a higher permeability (scEBM R-OGD: 128.7 ± 14.3%) in comparison with the control (scEBM R-Normoxia: 100 ± 5.8%) after reoxygenation, and scCM treatment reverted the OGD-induced barrier leakiness (scCM R-OGD: 98.5 ± 4.9%) (Fig. 5a). WB analysis revealed that scCM upregulated occludin (120.3% [107.5–123.8]), ZO-1 (123.2% [107.7–168.5]), and tricellulin (120.1% [109.8–133.7]) expression (Fig. 5b). Besides, IF analysis suggested that scCM treatment preserved the TJ distribution at the cell boundaries (Fig. 5c). Interestingly, the VEGFR2 phosphorylation was increased in scCM-treated CMECs, with no changes detected in ERK1/2 nor AKT activation (Fig. 5d). Besides, scCM induced the expression of VCAM-1, ICAM-1, and COX2 in CMECs during reoxygenation (Fig. 5d).

The article "Secretome of endothelial progenitor cells from stroke patients promotes endothelial barrier tightness and protects against hypoxia-induced vascular leakage" was retracted in 2024. Reason: errors in the cell lines or tissues.

**Fig. 5:** OGD-induced vascular leakage in vitro is prevented by scCM. Treatment with scCM during reoxygenation (24 h) abolished the OGD-induced increase in permeability on CMECs (**a**). WB analysis revealed that scCM increased occludin, ZO-1, and tricellulin expression (**b**) and favoured their localization at cell junctions (**c**). scCM increased VEGFR2 activation, while it did not affect ERK1/2 or AKT activation (**d**). Besides, scCM upregulated VCAM-1, ICAM-1, and COX2 expression (**d**). Data represent median (interquartile range) [**b** and **d**] or mean ± SD [**a**] (*n* = 3–5). *P < 0.05 vs scEBM; $*P* < 0.05 vs R-OGD scEBM. Scale bar: 10 μm

In BLECs, OGD exposure increased the permeability after reoxygenation (scEBM R-normoxia: 100 ± 5.9% vs scEBM R-OGD: 125.8 ± 14.3%) and scCM prevented the OGD-induced leakiness (scCM R-OGD: 96.1 ± 15.4%) (Fig. 6a). Such effect is possibly associated with the upregulation of claudin 5 (154.2% [106.9–224.7]) (Fig. 6b) and the restoration of TJ localization/assembly (Fig. 6c). Oppositely to the effects in CMECs, scCM inhibited both VEGFR2 and ERK1/2 activation, while it had no effect in the expression of VCAM-1, ICAM-1, and COX2 under OGD conditions (Fig. 6d).

**Fig. 6:** OGD-induced in vitro BBB leakage is prevented by scCM. Treatment with scCM during reoxygenation (24 h) abolished the OGD-induced increase in permeability on BLECs (**a**). WB analysis revealed that scCM increased claudin 5 expression (**b**) and favoured its localization at the cell junctions (**c**). scCM decreased VEGFR2 and ERK1/2 activation during reoxygenation (**d**). Moreover, scCM increased ICAM-1 expression in normoxic conditions but had no effect on BLECs exposed to OGD (**d**). Data represent median (interquartile range) [**b** and **d**] or mean ± SD [**a**] (*n* = 3–5). *P < 0.05 vs scEBM; $*P* < 0.5 vs R-OGD scEBM. Scale bar: 10 μm

### scCM prevents TNFα-induced BBB leakage

The exacerbation of TNFα production by perivascular cells plays a key role in neuroinflammation and vascular leakage after stroke [32]. Since scCM had a protective effect in the vascular barrier under hypoxic conditions, we investigated whether it was also able to prevent the TNFα-induced barrier breakdown. In CMECs, TNFα did not significantly affect the permeability (Additional file 18: Figure S16a). On the other hand, TNFα induced a drastic elevation of BLECs permeability (scEBM control: 101.4% [93.3–106] vs scEBM TNFα 473% [375.2–1049.1]) and scCM partially prevented the BBB leakage (245.8% [202.9–688.3]) (Additional file 18: Figure S16b). In parallel, TNFα treatment downregulated occludin expression (scEBM control: 100 ± 32.5% vs scEBM TNFα: 39.2 ± 9.5%) and pre-treatment with scCM partially inhibited (scCM TNFα: 64.8 ± 25.7%) this effect in BLECs (Additional file 18: Figure S16c).

The article "Secretome of endothelial progenitor cells from stroke patients promotes endothelial barrier tightness and protects against hypoxia-induced vascular leakage" was retracted in 2024. Reason: errors in the cell lines or tissues.

## Discussion

Ischemic stroke is a major cause of death and disability worldwide, and the current therapeutic interventions targeting brain repair are still scarce. Over the last years, cell therapy with EPCs has been pinpointed as a promising approach for the enhancement of both vascular remodelling and neurogenesis after stroke [8, 9, 33]. However, concerns associated with cell-based therapies have limited their application for clinical purposes. In this context, cell-free therapies have been considered as an interesting alternative and some studies have reported beneficial effects of EPC-secretome in pre-clinical models of stroke and hypoperfusion [14, 15]. The present study reports a reproducible method for high-scale production of EPC-secretome (scCM) for therapeutic purposes. Further, we investigated the effect of scCM in primary human ECs, with a particular focus on angiogenesis and the regulation of vascular permeability (Fig. 7a). Overall, our results suggested that scCM exhibits an important angiogenic activity while lacking the negative effects of VEGF-A on vascular barrier properties. To the best of our knowledge, this is the first study evaluating the effect of EPC-secretome produced under high-scale conditions in a human in vitro BBB model. The results from this study expand the current knowledge about the mechanisms underlying the EPC-mediated effects on vascular cells and highlight proteins/pathways, which can be targeted for the simultaneous promotion of angiogenesis and vascular protection in the brain (Fig. 7b).

**Fig. 7:** Network map of potential proteins/pathways involved in scCM-induced effects. (**a**) Schematic overview of angiogenesis process and in vitro assays proposed for evaluating EPC-secretome effects. Human CD34^+^-derived cord-blood hematopoietic endothelial cells (CD34^+^-ECs) were used to study angiogenesis (proliferation, cell migration, and tubulogenesis). To investigate mechanisms involved in vascular maturation, CD34^+^-EC were seeded on the surface of Matrigel™-coated Transwell inserts and cultivated in monocultures (CMECs). Finally, to study the effect of EPC-secretome on brain capillaries, we used an in vitro BBB model which consisted in seeding CD34^+^-ECs on Matrigel™-coated Transwell inserts and co-cultivating them with human brain pericytes, which enabled CD34^+^-ECs to acquire a brain-like endothelial cell phenotype (BLECs). (**b**) Proteins present in scCM were converted in gene identifiers and were then grouped according to their biological function/pathway (metabolic pathways, growth factors, inflammatory response, basal membrane (BM) regulation, cytoskeletal regulation, and integrin pathway). An interaction network was prepared using the Cytoscape software (version 3.8.2, released 2020.10.24). The regulation of MAPK activity might play an essential role in the scCM-induced angiogenesis in human primary ECs. In parallel, scCM promotes vascular maturation of newly formed vessels and protects the BBB integrity under ischemic and inflammatory conditions

Initially, we have compared the angiogenic activity of the secretome produced by EPCs derived from SP and HD obtained by LSP. Although accumulating evidence has suggested that cardiovascular risk factors are associated with dysfunction and a reduced number of EPCs [34–37], the influence of cerebrovascular diseases on circulating EPCs is still debated. For instance, studies have shown that stroke was associated with a reduced number of circulating EPCs [38] and impairment of EPC function [39, 40]. On the other hand, some studies have also reported an increase in the number of circulating EPCs in stroke patients [16, 41]. Additionally, pre-clinical studies have shown that focal cerebral ischemia promotes EPCs mobilization and enhances the tubulogenesis of EPCs in vitro [10]. Besides, hypoxic pre-conditioning of EPCs has been proposed as a strategy to enhance their angiogenic properties [42]. In a nutshell, such studies have suggested that ischemia might improve the angiogenic abilities of EPCs and enhance therapeutic outcomes. Our in vitro studies (proliferation, migration, and tubulogenesis) have not found any difference in the angiogenic properties of EPC-secretome from stroke and healthy donors. Therefore, the use of autologous EPCs from stroke patients might be the alternative for secretome production, as this approach would shorten ethical approvals. From our point of view, this study is a first step towards developing cell-based but cell-free formulations obtained under optimized GMP conditions for future clinical applications.

The article "Secretome of endothelial progenitor cells from stroke patients promotes endothelial barrier tightness and protects against hypoxia-induced vascular leakage" was retracted in 2024. Reason: errors in the cell lines or tissues.

The EPC-secretome obtained under HSP conditions (scCM) showed a higher protein concentration (168-fold increase) in comparison with LSP. Additionally, the composition of LSP and HSP might be slightly different, since we observed a consistent effect of high-scale produced EPC-secretome on tubulogenesis, while the secretome produced under LSP had no effect. It is important to highlight that the standardization of HSP of EPC-secretome consisted in several challenging steps, such as controlling cell density at seeding, change of medium, and concentration of large volumes of conditioned medium. Therefore, further studies are necessary to understand the difference on composition of the secretome produced under low- and high-scale conditions; however, we consider it is an important step towards developing cell-based therapies for stroke treatment.

Proteome profiler analysis revealed an equitable presence of key angiogenesis-related proteins in two scCM batches, indicating low batch-to-batch variation under HSP conditions. Further, DDA-MS analysis of scCM revealed an overrepresentation of proteins associated with the modulation of cell metabolism, which is in agreement with previous studies reporting that the beneficial effects of cell therapy are due, at least in part, to metabolism regulation of injured cells [43–45]. Indeed, the delivery of key proteins involved in the regulation of glycolysis, pyruvate, and pentose phosphate pathways by EPC-secretome might boost cell metabolism or rescue metabolic activity in ischemic-injured cells. Additionally, the enrichment of proteins participating in cell cycle and cytoskeleton regulation might contribute to the scCM-induced promotion of CD34^+^-ECs proliferation, migration, and tubulogenesis, which were similar to the effects induced by VEGF-A, a key regulator of angiogenesis. The scCM-induced angiogenesis was partially mediated through MAPK activation, whereas PI3K/AKT pathway might not play a major role on this process. Our results are partially different from a previous study reporting that AKT is the main pathway underlying EPC-secretome-induced angiogenesis in rat immortalized brain ECs, while ERK activation plays a minor role in this process [46]. The RTK activation by growth factors might be the key event leading to downstream MAPK activation since the inhibition of both VEGFR2 and FGFR completely abolished scCM-induced angiogenesis. The presence of growth factors and adapter molecules on scCM possibly contribute to RTK/MAPK activation. Additionally, the presence of integrin ligands in scCM might contribute to VEGFR2/ERK activation, given that integrins can increase the efficiency of RTK activation [47] and the coupling between upstream and downstream events in the RTK-Ras-MAPK cascade [48]. Besides, the crosstalk between VEGFR and integrin receptors is necessary to induce the VEGFR2-mediated angiogenesis [49]. In summary, our results suggest that the coordinated action of growth factors, adapter molecules, and integrin ligands plays a pivotal role in scCM-induced angiogenesis (Fig. 7b).

The article "Secretome of endothelial progenitor cells from stroke patients promotes endothelial barrier tightness and protects against hypoxia-induced vascular leakage" was retracted in 2024. Reason: errors in the cell lines or tissues.

Vascular leakage following acute stroke is a major hazard that can compromise brain function as well as the therapeutic outcomes of treatments targeting brain repair. Considering that the local production of VEGF-A is critical for vascular disruption following stroke [50], we investigated the effect of scCM on permeability using an in vitro model of newly formed vessels (CMECs) and an already established BBB model in vitro (BLECs). As expected, VEGF-A evoked barrier leakage, while scCM promoted a consistent decrease in CMECs permeability together with an upregulation of junctional proteins. Interestingly, scCM upregulated P-gp expression in BLECs, suggesting that it might potentiate the transport of xenobiotics out of the brain through the BBB. Further, mRNA sequencing analysis of CMECs revealed that scCM upregulated the expression of several IFN-related genes. This finding is in accord with the presence of several proteins related to inflammatory pathways detected in scCM by MS analysis. Among them, STAT1 can translocate to the nucleus and activate the transcription of IFN-stimulated genes [51], while NMI, ISG15, and HMGB1 are IFN-induced proteins [52–54] (Fig. 7b). A body of evidence has highlighted a potential beneficial effect of the IFN pathway on the regulation of vessel maturation and inflammatory response. In this regard, IFN can stabilize barrier properties of in vitro BBB models [55] and act as a modulator of cytokine networks, reducing the cytokine-induced neutrophil infiltration and attenuating BBB disruption [56, 57]. Besides, IFN-β might counteract the TJ disruption induced by the inflammatory response on brain ECs [56]. Such findings are in agreement with the protective effect of scCM against TNFα-induced disruption in BLECs. In parallel, our results suggest that scCM-induced barrier tightness is mediated through a moderate downregulation of Wnt activation, as highlighted by a decrease in active β-catenin content. Interestingly, some studies have reported evidence showing a common modulation of the Wnt and IFN pathways in the regulation of inflammatory responses. For instance, members of the miR-34 family, which are well-known repressors of Wnt/β-catenin signalling, potentiate the induction of IFN-responsive genes and their signalling pathways [58]. Another study has shown that PEGylated-IFN inhibited β-catenin translocation to the nucleus and Wnt signalling in hepatoma cell lines [59]. Overall, our results suggest that the orchestrated modulation of the Wnt pathway and IFN signalling could be an underlying mechanism involved in scCM-induced barrier tightness under physiological conditions.

The article "Secretome of endothelial progenitor cells from stroke patients promotes endothelial barrier tightness and protects against hypoxia-induced vascular leakage" was retracted in 2024. Reason: errors in the cell lines or tissues.

Next, we tested the potential beneficial effect of scCM on cells exposed to hypoxic conditions. In this regard, treatment with scCM completely abolished the OGD-induced leakage on CMECs and BLECs. This effect was possibly mediated through the regulation of junctional proteins expression and localization, leading to vascular protection against hypoxic-induced injury. The activity of integrin ligands and modulators of the extra-cellular matrix might be involved in scCM-mediated protection in OGD conditions since the degradation of the basal membrane involving the BBB is directly associated with ischemia-induced vascular disruption [60]. A potential activation of the IFN pathway by scCM also might contribute to the scCM-mediated vascular protection under ischemic conditions. Besides, the presence of small levels of growth factors in EPC-secretome might have a protective effect on injured cells, given that growth factors can promote anti-apoptotic effects [61]. Indeed, scCM increased VEGFR2 activation on CMECs exposed to OGD conditions. In parallel, scCM upregulated the expression of adhesion molecules (VCAM-1 and ICAM-1) and COX2, known molecular targets of VEGF pathway activation [62, 63]. Besides, the enrichment of proteins involved in inflammatory responses might contribute to the scCM-induced upregulation of adhesion molecules (Fig. 7b). VCAM-1 is important to promote close intercellular adhesion between ECs and pericytes, and it is required for blood vessel formation [64]. Besides, COX-2 plays a pivotal role in the VEGF-induced angiogenesis [65]. The scCM-induced adhesion molecule upregulation might favour the homing of leukocytes and circulating EPCs on injured vessels, which can further potentiate angiogenesis. On the other hand, the scCM-induced downregulation of VEGFR2 and ERK1/2 activation in BLECs exposed to OGD conditions might have a beneficial effect, considering that hypoxia-driven VEGF-A production is the main mechanism inducing BBB leakage [50] and that MAPK activation plays a key role in vascular injury induced by ischemia [66, 67]. Altogether, these results suggest that scCM can prevent the hypoxia-induced vascular leakiness, protecting the brain from edema-related deleterious effects.

The article "Secretome of endothelial progenitor cells from stroke patients promotes endothelial barrier tightness and protects against hypoxia-induced vascular leakage" was retracted in 2024. Reason: errors in the cell lines or tissues.

Altogether, our results suggest that the scCM-elicited effects in proliferative and quiescent ECs were mediated through an orchestrated action of growth factors, integrin ligands, inflammatory mediators, enzymes regulating cell metabolism, and proteins regulating cytoskeleton and basement membrane composition (Fig. 7b). The regulation of the MAPK pathway seems to be a key component of scCM-driven effects since a variety of proteins identified are directly linked to ERK1/2 activation and the scCM-treatment leads to the activation and/or inhibition of MAPK. However, other molecules present in the EPCs secretome, such as lipids and microRNAs, should be also considered but not addressed in this study. Certainly, further studies are necessary to better understand the mechanisms of EPC-secretome actions and identify the key molecules triggering its beneficial effects. It is noteworthy that we have used for this study cryopreserved EPCs obtained from freshly isolated PBMCs. Despite the fact that the effect of cryopreservation on EPCs’ physiology is still controversial [68–70], such strategy allows the creation of a bank of EPCs from different donors or sources (e.g. bone marrow, blood, umbilical cord) for screening the cells with better angiogenic activity. We consider that a potential effect of cryopreservation needs to be taken into account for future studies in order to optimize EPC-secretome use as a therapeutic alternative for promoting brain angiogenesis and neurorepair. However, our study provides valuable information to understand the underlying mechanisms of EPC-mediated effects to develop cell-based therapies for stroke.

## Conclusions

Herein, we describe a reproducible method for a high-scale production of EPC-secretome and report pre-clinical evidence supporting its potential benefits for regenerative medicine. In particular, our results using human primary ECs suggest that scCM boosts angiogenesis-related processes while preserving the vascular barrier function in healthy vessels. In addition, scCM might promote vessel maturation and restore/preserve the BBB function in ischemic or inflammatory conditions. In conclusion, our results pave the way for future clinical trials employing EPC-secretome in order to promote brain repair after stroke.

## Supplementary Information

**Additional file 1: Figure S1.** scCM increases CD34^+^-ECs proliferation. scHD-CM, scSP-CM, and scCM (batch 1 and 2) increase ATP production by CD34^+^-ECs. Data represent median (interquartile range) (*n* = 3–7), *P < 0.05 vs scEBM.

**Additional file 2: Figure S2** Effect of scCM treatment in the endothelial barrier properties. The permeability for radiolabelled-sucrose is enhanced in CMECs compared with BLECs (**a**). VEGF-A (50 ng/mL) induced vascular leakage in both CMECs and BLECs (**b**). Representative images of immunofluorescence performed in CMECs (**c**) and BLECs (**d**) for detection of claudin 5, ZO-1, occludin, and VE-cadherin. Data represent median (interquartile range) (*n* = 3–5). Scale bar: 10 μm.

The article "Secretome of endothelial progenitor cells from stroke patients promotes endothelial barrier tightness and protects against hypoxia-induced vascular leakage" was retracted in 2024. Reason: errors in the cell lines or tissues.

**Additional file 3: Figure S3.** Representative images of pilot experiments performed to test the antibodies used in the study. Black arrows show the corresponding bands for every antibody according to the molecular weight predicted by the manufacturer. (**a**) phospho-AKT and pan-AKT; (**b**) phospho-VEGFR2 and pan-VEGFR2; (**c**) phospho-ERK1/2 and pan-ERK 1/2; (**d**) non-phospho-β-catenin and pan- β-catenin; (**e**) ABCA1; (**f**) BCRP; (**g**) P-gp; (**h**) COX-2; (**i**) VCAM-1; (**j**) ICAM-1; (**k**) claudin 5; (**l**) VE-cadherin; (**m**) occludin; (**n**) ZO-1; (**o**) tricellulin; (**p**) claudin 3. For images **A**–**D**, membranes were firstly probed with phospho-antibodies and then reprobed with pan-antibodies.

**Additional file 4: Figure S4.** Images used for western blotting analysis of ERK1/2, AKT, and VEGFR2 phosphorylation in proliferative CD34^+^-EC in response to acute administration (0–60 min) of scCM (5 μg/mL) (Fig. 3a). bFGF (basic FGF) represented in (**a**) was not considered for analysis.

**Additional file 5: Figure S5.** Images used for western blotting analysis of ERK1/2, AKT, and VEGFR2 phosphorylation in proliferative CD34^+^-EC in response to administration (4 or 24 h) of scCM (5 μg/mL) (Figure 3b).

**Additional file 6: Figure S6.** Images used for western blotting analysis of ZO-1, VE-cadherin, occludin, claudin 5, claudin 3, non-phospho-catenin, and pan-catenin in CMECs in response to administration (48 h) of scCM (5 μg/mL) (Fig. 4b and e). scCM-1: batch 1; scCM-2: batch 2. Analysis of scCM-2 were not presented in the manuscript.

**Additional file 7: Figure S7.** Images used for western blotting analysis of ZO-1, VE-cadherin, occludin, and claudin 5 in BLECs in response to administration (48 h) of scCM (5 μg/mL) (Fig. 4b). scCM-1: batch 1; scCM-2: batch 2. Analysis of scCM-2 were not presented in the manuscript.

**Additional file 8: Figure S8.** Images used for western blotting analysis claudin 5, tricellulin, VEGFR2, VCAM-1, COX-2, occludin, VE-Cadherin, ZO-1, and ERK1/2 in CMECs exposed to normoxic (N) or OGD conditions and reoxygenation (R-N-scEBM; R-N-scCM; R-OGD-scEBM; R-OGD-scCM) (Fig. 5 and Additional file 17: Figure S15).

**Additional file 9: Figure S9.** Images used for western blotting analysis of claudin 5, ZO-1, VE-cadherin, VEGFR2, VCAM, AKT, ERK1/2, and occludin in CMECs exposed to normoxic (N) or OGD conditions and reoxygenation (R-N-scEBM; R-N-scCM; R-OGD-scEBM; R-OGD-scCM) (Fig. 5 and Additional file 17: Figure S15).

The article "Secretome of endothelial progenitor cells from stroke patients promotes endothelial barrier tightness and protects against hypoxia-induced vascular leakage" was retracted in 2024. Reason: errors in the cell lines or tissues.

**Additional file 10: Figure S10.** Images used for western blotting analysis of VEGFR2, claudin 5, ZO-1, VE-cadherin, occludin, ICAM-1, AKT, ERK1/2, tricellulin, VCAM-1, and COX2 in BLECs exposed to normoxic (N) or OGD conditions and reoxygenation (R-N-scEBM; R-N-scCM; R-OGD-scEBM; R-OGD-scCM) (Fig. 6 and Additional file 17: Figure S15).

**Additional file 11: Figure S11.** Images used for western blotting analysis of VEGFR2, occludin, VE-cadherin, ZO-1, claudin 5, ERK1/2, AKT, and ICAM-1 in BLECs exposed to normoxic (N) or OGD conditions and reoxygenation (R-N-scEBM; R-N-scCM; R-OGD-scEBM; R-OGD-scCM) (Fig. 6 and Additional file 17: Figure S15).

**Additional file 12: Figure S12.** Images used for western blotting analysis of ABCA1, BCRP, and P-gp in CMECs (**a**–**c**) and BLECs (**d**–**e**) in response to administration (48 h) of scCM (5 μg/mL) (Additional file 15: Figure S14d). scCM-1: batch 1; scCM-2: batch 2. Analysis of scCM-2 were not presented in the manuscript.

**Additional file 13: Figure S13.** Images used for western blotting analysis of claudin 5, ZO-1, occludin, and VE-cadherin in BLECs treated with vehicle or TNFα (10 ng/mL) (Additional file 18: Figure S5c).

**Additional file 14: Table S1.**

**Additional file 15: Figure S14.** Effect of scCM treatment in the endothelial barrier properties. Co-staining with phalloidin and ZO-1 suggests that scCM promotes the accumulation of actin fibres at the cell borders (yellow arrowheads) and decreases its distribution across the cytoplasm of CMECs (**a**) and BLECs (**b**). scCM upregulates P-gp expression on BLECs, whereas it did not affect ABCA1 and BCRP expression (**c**). Data represent median (interquartile range) (*n* = 4–8). *P < 0.05 vs scEBM. Scale bar: 10 μm.

**Additional file 16: Table S2.**

**Additional file 17: Figure S15.** Effect of oxygen–glucose deprivation (OGD) on *in vitro* vascular permeability. OGD (6 h) had no effect on permeability of CMECs (**a**), while it induced vascular leakage in BLECs (**b**). OGD upregulated the mRNA expression of target genes, such as HIF1A, VEGF-A, and Glut-1 (**c**). Western blot analysis did not show a marked effect of OGD on the expression of junctional proteins (**d**); however, IF analysis suggested that OGD induces their accumulation in the cytoplasm (**e**). Data represent median (interquartile range) (*n* = 3–4). *P < 0.05 vs scEBM. Scale bar: 10 μm.

**Additional file 18: Figure S16.** Effect of TNFα on *in vitro* vascular permeability. CMECs and BLECs were pre-treated (24 h) with scEBM or scCM (5 μ/mL) and then TNFα (10 ng/mL) was administered to the cells. Whereas TNFα had no significant effect on permeability of CMECs (**a**), scCM partially prevented TNFα-induced leakage in BLECs (**b**). WB analysis showed that scCM partially restored the TNFα-induced downregulation of occludin in BLECs (**c**). Data represent median (interquartile range) [a and b] or mean ± SD [c] (*n* = 4–8). *P < 0.05 vs scEBM control.

The article "Secretome of endothelial progenitor cells from stroke patients promotes endothelial barrier tightness and protects against hypoxia-induced vascular leakage" was retracted in 2024. Reason: errors in the cell lines or tissues.

## Data Availability

The datasets used and/or analysed during this study are available from the corresponding authors upon reasonable request.

## Abbreviations

AJ: Adherens junctions
AKT: Protein kinase B
ATP: Adenosine triphosphate
BBB: Blood–brain barrier
BLEC: Brain-like endothelial cells
BSA: Bovine serum albumin
CD34 + -EC: CD34 +-derived cord-blood hematopoietic endothelial cells
CM: Conditioned medium
CMEC: Confluent monolayer of endothelial cells
CNS: Central nervous system
COX-2: Cyclooxygenase 2
DTT: Dithiothreitol
ECGS: Endothelial cell growth supplement
EPC: Endothelial progenitor cells
ECM: Endothelial cell medium
EGM: Endothelial growth medium
ERK1/2: Extracellular signal-regulated kinase ½
HBP: Human brain pericytes
HD: Healthy donor
hFN: Human fibronectin
HSP: High-scale production
HIF1α: Hypoxia-induced factor 1α
ICAM-1: Intercellular adhesion molecule 1
IFN: Interferon
LSP: Low-scale production
MAPK: Mitogen-activated protein kinase
Min: Minutes
MMP9: Metalloproteinase 9
MS: Mass spectrometry
Naf: Sodium fluorescein
NGS: Normal goat serum
OGD: Oxygen–glucose deprivation
PBS-CMF: Phosphate-buffered saline calcium magnesium-free
PDGF: Platelet-derived growth factor
Pe: Permeability coefficient
qRT-PCR: Real-time quantitative reverse transcription polymerase chain reaction
RH: Ringer-Hepes buffer
RT: Room temperature
RTK: Receptor tyrosine kinase
scCM: Super-concentrated conditioned medium
SP: Stroke patient
TIMP1/4: Tissue inhibitor of metalloproteinase 1 and 4
TJ: Tight junction
VCAM-1: Vascular cell adhesion molecule 1
VEGF-A: Vascular endothelial cell growth factor A
VEGFR2: VEGF receptor 2
uPA: Urokinase-type plasminogen activator
WB: Western blot
